The article "Protective effects of calcium gluconate on osteoarthritis induced by anterior cruciate ligament transection and partial medial meniscectomy in Sprague–Dawley rats" was published in 2014. Journal: J Orthop Surg Res.

# Protective effects of calcium gluconate on osteoarthritis induced by anterior cruciate ligament transection and partial medial meniscectomy in Sprague–Dawley rats

**DOI:** 10.1186/1749-799X-9-14

**Published:** 2014-03-07

**Authors:** Su-Jin Kang, Joo-Wan Kim, Ki-Young Kim, Sae-Kwang Ku, Young-Joon Lee

**Affiliations:** 1 The Medical Research Center for Globalization of Herbal Medicine, Daegu Haany University, Gyeongsan, Gyeongsangbuk-do 712-715, Repulic of Korea; 2 Department of Preventive Medicine, College of Korean Medicine, Deagu Haany University, 1, Hannydaero, Gyeongsan, Gyeongsangbuk-do 712-715, Republic of Korea; 3 Glucan Corporation and Marine Bio-Industry Development Center, Busan 619-912, Republic of Korea; 4 Department of Histology and Anatomy, College of Korean Medicine, Daegu Haany University, 1, Hannydaero, Gyeongsan, Gyeongsangbuk-do 712-715, Republic of Korea

**Keywords:** Calcium gluconate, Osteoarthritis, COX-2, Apoptosis

## Abstract

**Background:**

This study aimed to determine whether calcium gluconate exerts protective effects on osteoarthritis (OA) induced by anterior cruciate ligament (ACL) transection and partial medial meniscectomy.

**Methods:**

Calcium gluconate was administered by mouth daily for 84 days to male ACL transected and partial medial meniscectomized Sprague–Dawley rats 1 week after operation.

**Results:**

Eighty-four days of treatment with 50 mg/kg calcium gluconate led to a lower degree of articular stiffness and cartilage damage compared to the OA control, possibly through inhibition of overexpressed cyclooxygenase (COX)-2 and related chondrocyte apoptosis. Similar favorable effects on stiffness and cartilage were detected in calcium gluconate-administered rats. Additionally, calcium gluconate increased 5-bromo-2′-deoxyuridine (BrdU) uptake based on observation of BrdU-immunoreactive cells on both the femur and tibia articular surface cartilages 84 days after intra-joint treatment with calcium gluconate.

**Conclusions:**

Taken together, our results demonstrate that calcium gluconate has a protective effect against OA through inhibition of COX-2 and related chondrocyte apoptosis.

## Background

Osteoarthritis (OA) is characterized by changes in the structure and function of the articulation. OA is a degenerative process that takes place in the articular cartilage [1], which has a highly limited capacity to regenerate and repair due to its avascular nature. Chondrocytes are a pivotal component of the pathogenesis of OA. Under normal conditions, the synthetic and catabolic activities of chondrocytes are balanced to maintain the integrity of articular cartilage *in vivo*. Stimuli, such as nitric oxide, prostaglandin E2, Fas ligand, and tumor necrosis factor-α [2-5], disrupt the ability of chondrocytes to maintain the integrity of articular cartilage, leading ultimately to apoptosis. Apoptosis of chondrocytes was initially reported in relation to the differentiation of hypertrophic chondrocytes and ossification of the growth plate [6,7]. Thus, modulation of the mechanism(s) of apoptosis-inducing factors is considered a novel strategy for the treatment of OA [8].

Caspase-3 is one of the key mediators of apoptosis, as it is either partially or totally responsible for the proteolytic cleavage of many key proteins, such as nuclear enzyme poly-ADP ribose polymerase (PARP) [9]. PARP is a representative target molecule of caspase-3 that facilitates activation of the DNA repair system by caspase-mediated cleavage [10,11].

Prostaglandin is involved in the pathogenesis of OA [3]. It is derived primarily from cyclooxygenase (COX)-2 and plays a role as a key mediator of the inflammation and pain associated with OA. Conversely, inhibition of COX-2 and prostaglandin synthesis by traditional non-steroidal anti-inflammatory drugs (NSAIDs) and COX-2 inhibitors ameliorate OA symptoms [12,13].

Accumulating evidence suggests that calcium salts possess anti-inflammatory activity. Calcium chloride has been advocated for the treatment of urticaria, acute edema, pruritis, and erythema [14]; calcium carbonate and calcium gluconate have been used for the treatment of insect stings [15], and calcium hydroxide has been used to suppress periapical inflammation in dental practice [16]. Thus, we examined whether calcium gluconate exerts protective effects on OA induced by anterior cruciate ligament (ACL) transection and partial medial meniscectomy.

## Methods

### Animals and husbandry

Thirty-six male Sprague–Dawley rats (160–180 g, 6 weeks old upon receipt, SLC, Osaka, Japan) were housed (3–4 per cage) and allowed to acclimate 9 days before use (light/dark cycle, 12 h). A normal rodent pellet diet and water were supplied *ad libitum* throughout all experiments, including during acclimatization. All animals were fasted overnight prior to sacrifice (approximately 18 h with *ad libitum* access to water) and treated according to the Guide for the Care and Use of Laboratory Animals of the Institute of Laboratory Animal Resources, Commission on Life Science, 1996 National Research Council, Washington D.C.

### Preparations and administration of test materials

In sham control rats, distilled water (5 ml/kg) was orally administered daily. In OA control rats, animals were orally administered 1 ml/kg distilled water in the absence of calcium gluconate. As a reference control, 2 mg/kg diclofenac sodium (Sigma, St. Louis, MO, USA) dissolved in saline was administered subcutaneously daily for 84 days beginning 1 week after induction of OA. Calcium gluconate (25, 50, and 100 mg/kg) was dissolved in distilled water and orally administered daily for 84 days (5 ml/kg) to OA rats that underwent ACL transection and partial medial meniscectomy, beginning 1 week after the operation.

### Induction of OA

Rats were anesthetized with an intraperitoneal injection (25 mg/kg) of Zoletile mixture (Zoletile 50, Virbac Lab., Carros Cedex, France). The surgery was carried out according to the method of Kamekura et al. [17]. Briefly, the OA treatment group underwent open surgery involving ACL transection and partial medial meniscectomy via an incision in the medial aspect of the joint capsule, anterior to the medial collateral ligament. The operation was performed using a 15° 5-mm blade micro-surgical knife, micro-iris scissors, and micro-corneal suturing forceps and #11 and #15 blades. Following surgery, saline was used for washing tissue debris; the incision was closed in two layers. The joint capsule was sutured independently from peripheral tissues using dissolvable 5–0 Vicryl sutures, and the skin was closed by interrupted sutures using silk. This treatment was used to induce OA pathogenesis and referred to as operated-induced sides. Conversely, the right (non-operated intact side) knee joint was used as the contralateral treatment. The second group of rats underwent a sham operation in which a similar incision in the joint capsule was made, but ACL transection and partial medial meniscectomy were not performed. Only the left knees of sham animals were used as controls for disease progression.

### Evaluation of clinical symptom changes

Body weights were measured weekly from the start of calcium gluconate treatment until sacrifice with an automatic electronic balance (Precisa Instrument, Dietikon, Switzerland). In addition, body weight gain during 12 weeks of observation (following calcium gluconate or diclofenac sodium treatments) was calculated. The thickness of OA in the hind knee (right side) was measured using an electronic digital caliper (Mitutoyo, Kawasaki, Japan) and recorded weekly following treatment. OA-operated knees in all animals were dissected from the coxofemoral region to the ankle, leaving the articular capsule intact. After dissection, the maximum extension angle of each knee was measured, with 0° corresponding to the maximum possible extension.

### Histology and evaluation

Portions of the knee joints were sampled in a manner that preserved the joint capsule and fixed in 10% neutral-buffered formalin. After 5 days of fixation, sections were decalcified using a decalcifying solution (24.4% formic acid, 0.5 N sodium hydroxide) for 5 days (mixed decalcifying solution was exchanged daily for 5 days). Median joint parts were then longitudinally trimmed and embedded in paraffin, sectioned (3–4 μm), and stained with hematoxylin and eosin (H&E) or Safranin O for cartilage. Articular cartilage injuries found in the knees of rats were evaluated and recorded using the Mankin score, as referred to by Armstrong et al. [18] and Lovász et al. [19]. Tibial and femoral articular cartilage thicknesses were measured by means of histomorphometric analyses in longitudinally trimmed samples at the micrometer level using a digital image analyzer (DMI-300, DMI, Daegu, Korea).

### BrdU uptake

Proliferating cells were labeled by means of an intraperitoneal injection of 5-bromo-2′-deoxyuridine (BrdU). One hour prior to injection of diclofenac sodium or oral administration of calcium gluconate (day 82 of treatment), rats received intraperitoneal injections of BrdU (MP Biomedicals, Solon, OH, USA; 50 mg/kg), in a volume of 2 ml/kg, dissolved in saline; the animals were sacrificed 72 h later. BrdU uptake was evaluated by immunohistochemistry using an anti-BrdU antibody.

### Immunohistochemical determination of apoptosis

To assess the effects of calcium gluconate on chondrocyte apoptosis within rat knees, the number of caspase-3-, PARP- and COX-2-positive cells were determined using immunohistochemistry. Fixed tissues were prepared, deparaffinized, and sectioned as described above histology part. After blocking for 1 h, sections were incubated with the appropriate primary antibody overnight at 4°C. They were incubated for 1 h with a biotinylated universal secondary antibody (Vector Lab. Inc., Burlingame, CA, USA; dilution 1:50) and then were incubated for 1 h with the ABC reagents (Vectastain Elite ABC kit, Vector Lab. Inc.; dilution 1:50). They were incubated in peroxidase substrate reagents (Vector Lab. Inc.), counterstained with Mayer's hematoxylin solution and observed under a light microscope (Nikon, Tokyo, Japan).

### Statistical analyses

Multiple comparison tests for the dosage groups were conducted. Data were subjected to one-way analysis of variance (ANOVA) or the non-parametric Kruskal–Wallis H comparison test, according to the results of the variance homogeneity Levene test. Statistical analyses were conducted using SPSS for Windows (Release 12.0 K, SPSS Inc., Chicago, IL, USA).

## Results

Knee thickness was increased significantly in OA-operated knees compared with sham control knees following treatment for 84 days. However, this increase in OA-induced knee thickness was decreased significantly compared with that in OA control knees 21 days after treatment with diclofenac sodium and 50 and 100 mg/kg calcium gluconate (Figure 1B).

**Figure 1:** **Body weight changes and knee thickness of OA rats. (A)** Body weight changes in OA rats following treatment with calcium gluconate. **(B)** Knee thickness in OA-induced joints was significantly (*p* < 0.01 or *p* < 0.05; arrow) decreased in calcium gluconate-treated rats compared with that in OA controls. Values represent the means ± standard deviation (SD) of eight rats. OA, osteoarthritis; AO, operation day; BT, 1 day before start of treatment; AT, start day of administration; AS, at sacrifice. All animals were fasted overnight prior to the start of administration and sacrifice.

Knee thickness of OA-operated joint capsule was increased significantly in all OA-induced groups compared with that in sham control rats. In contrast, diclofenac sodium and 50 and 100 mg/kg calcium gluconate treatment reduced knee thicknesses compared with those in OA controls (Table 1). The maximum extensor angles of induced knees at sacrifice in OA control rats were significantly greater (111.46%) compared with those in sham controls. However, these angles were significantly decreased by treatment with diclofenac sodium and 25, 50, and 100 mg/kg calcium gluconate compared with those in OA controls (Table 1).

**Table 1:** Knee thicknesses after joint capsule exposure and maximum extensor angles detected at sacrifice

**Groups**	**Knee thicknesses after joint capsule exposure at sacrifice (mm)**	**Maximum extensor angles (degrees)**
Controls		
Sham	7.72 ± 0.27	31.63 ± 3.46
OA	9.76 ± 0.60^a^	66.88 ± 7.47^a^
Diclofenac	9.16 ± 0.28^ac^	47.13 ± 7.26^ac^
Calcium gluconate-treated		
100 mg/kg	8.96 ± 0.40^ac^	39.50 ± 6.52^bc^
50 mg/kg	9.16 ± 0.20^ac^	47.38 ± 7.48^ac^
25 mg/kg	9.52 ± 0.64^a^	66.75 ± 10.33^a^

After 84 days of continuous oral treatment of calcium gluconate or subcutaneous treatment of diclofenac sodium in OA rats. Values are expressed as mean ± SD of eight rats. OA, osteoarthritis; ^a^*p* < 0.01 and ^b^*p* < 0.05 compared with sham control; ^c^*p* < 0.01 compared with OA control.

Total Mankin scores of induced femur and tibia articular cartilage in OA controls were significantly increased compared with those of the sham control; the scores in diclofenac sodium- and calcium gluconate (50 and 100 mg/kg)-treated groups were significantly decreased as compared with those in OA control, respectively (Table 2).

**Table 2:** Mankin scores detected in femur and tibia at sacrifice

**Groups**	**Femur**					**Tibia**				
	**Surface**	**Hypocellularity**	**Clones**	**Safranin O**	**Total**^**a**^	**Surface**	**Hypocellularity**	**Clones**	**Safranin O**	**Total**^**a**^
Controls										
Sham	0.25 ± 0.46	0.25 ± 0.46	0.00 ± 0.00	0.38 ± 0.52	0.88 ± 0.64	0.38 ± 0.52	0.38 ± 0.52	0.13 ± 0.35	0.38 ± 0.52	1.25 ± 1.39
OA	2.75 ± 0.46^b^	2.50 ± 0.53^a^	2.25 ± 0.89^b^	2.38 ± 0.52^b^	9.88 ± 1.13^b^	2.63 ± 0.52^b^	2.38 ± 0.52^b^	2.63 ± 0.52^b^	2.13 ± 0.83^b^	9.75 ± 1.04^b^
Diclofenac	2.00 ± 0.53^cd^	1.63 ± 0.52^bd^	2.25 ± 0.71^b^	1.38 ± 0.52^bd^	7.25 ± 1.39^bd^	1.88 ± 0.64^be^	1.63 ± 0.74^be^	1.75 ± 0.46^bd^	1.38 ± 0.74^ce^	6.63 ± 1.19^bd^
Calcium gluconate treated										
100 mg/kg	1.38 ± 0.74^bd^	1.25 ± 0.89^bd^	1.50 ± 0.76^b^	0.63 ± 0.52^d^	4.75 ± 1.98^bd^	1.25 ± 0.71^bd^	1.00 ± 0.76^d^	1.00 ± 0.76^bd^	1.25 ± 0.71^ce^	4.50 ± 2.20^bd^
50 mg/kg	2.00 ± 0.76^be^	1.50 ± 0.76^bd^	1.75 ± 0.46^b^	2.13 ± 0.35^b^	7.38 ± 1.77^bd^	2.00 ± 0.76^be^	1.63 ± 0.52^be^	1.50 ± 0.53^bd^	1.38 ± 0.74^ce^	6.50 ± 2.20^bd^
25 mg/kg	2.38 ± 0.74^b^	2.38 ± 0.52^b^	2.50 ± 0.53^b^	2.50 ± 0.76^b^	9.75 ± 1.16^b^	2.75 ± 0.46^b^	2.38 ± 0.74^b^	2.13 ± 0.64^b^	1.88 ± 0.83	9.13 ± 2.30^b^

After 84 days of continuous oral treatment of calcium gluconate or subcutaneous treatment of diclofenac sodium in OA rats. Values are expressed as mean ± SD of eight rats, scores (Table 1). OA, osteoarthritis. ^a^Total means Mankin score (max = 12); ^b^*p* < 0.01 and ^c^*p* < 0.05 compared with those of sham control; ^d^*p* < 0.01 and ^e^*p* < 0.05 compared with those of OA control.

OA-induced femur and tibia articular cartilage thicknesses decreased significantly in OA controls compared with sham controls but were significantly increased in the groups treated with diclofenac sodium and 50 and 100 mg/kg calcium gluconate, compared with those in the OA controls (Table 3 and Figure 2).With regard to the effects on cell proliferation, OA controls showed little or no BrdU staining in both the tibia and femur articular cartilage compared with sham controls. However, these decreases in BrdU-immunoreactive cells were significantly inhibited by treatment with 50 and 100 mg/kg calcium gluconate compared with OA controls (Figure 3).Caspase-3-immunoreactive cell numbers in OA-induced femur articular cartilage changed by 546.07% compared with those in the sham control, specifically, -34.09%, -62.26%, -28.52%, and -5.22% in the groups treated with diclofenac sodium and calcium gluconate (100, 50, and 25 mg/kg), respectively, compared with those in OA controls. Caspase-3-immunoreactive cell numbers in tibia articular cartilage changed by 452.83% compared with those in the sham control, specifically, -43.17%, -27.87%, -41.81%, and -5.46% in the groups treated with diclofenac sodium and calcium gluconate (100, 50, and 25 mg/kg), respectively, compared with those in the OA control (Figure 3). PARP-immunoreactive cell numbers in OA-induced femur articular cartilage thickness of OA controls changed by 485.37% compared with those in the sham control, specifically, -42.92%, -65.63%, -42.92%, and -0.42% in the groups treated with diclofenac sodium and calcium gluconate (100, 50, and 25 mg/kg), respectively, compared with those in the OA control. PARP-immunoreactive cell numbers in OA-induced tibia articular cartilage changed by 246.09% compared with those in the sham control, specifically, -41.21%, -59.30%, -38.19%, and -0.25% in the groups treated with diclofenac sodium and calcium gluconate (100, 50, and 25 mg/kg), respectively, compared with those in the OA control (Figure 3). COX-2-immunoreactive cell numbers in OA-induced femur articular cartilage thickness of OA controls changed by 287.86% compared with the sham control; specifically, -54.51%, -58.01%, -29.28%, and -0.92% in the groups treated with diclofenac sodium and calcium gluconate (100, 50, and 25 mg/kg), respectively, compared with those in the OA control. COX-2-immunoreactive cell numbers in OA-induced tibia articular cartilage changed by 253.90% compared with those in sham controls, specifically, -62.02%, -67.34%, -27.89%, and -2.02% in the groups treated with diclofenac sodium and calcium gluconate (100, 50, and 25 mg/kg), respectively, compared with those in the OA control (Figure 3).

**Table 3:** Histomorphometrical scores detected at sacrifice

**Groups**	**Thickness of articular cartilages**	
	**Femur**	**Tibia**
Controls		
Sham	570.69 ± 63.08	887.40 ± 75.03
OA	317.82 ± 77.79^a^	354.80 ± 46.41^a^
Diclofenac	472.56 ± 63.04^ab^	486.90 ± 41.78^ab^
Calcium gluconate treated		
100 mg/kg	574.06 ± 55.77^b^	689.43 ± 93.78^ab^
50 mg/kg	471.21 ± 47.69^ab^	482.43 ± 65.10^ab^
25 mg/kg	335.92 ± 40.20^a^	356.14 ± 52.71^a^

After 84 days continuous oral treatment of calcium gluconate or subcutaneous treatment of diclofenac sodium in OA rats. Values are expressed as mean ± SD of eight rats, μm; OA, osteoarthritis. ^a^*p* < 0.01 compared with sham control; ^b^*p* < 0.01 compared with OA control.

**Figure 2:** **Histopathological observations of the tibial and femoral articular cartilage.** Of sham controls **(A, B)**, OA controls **(C, D)**, and the diclofenac sodium **(E, F)** or calcium gluconate 100 mg/kg **(G, H)**, 50 mg/kg **(I, J),** and 25 mg/kg **(K, L)**-treated groups. Histopathological changes were markedly inhibited by calcium gluconate. Arrows indicate the thickness of tibia or femur articular cartilage; OA, osteoarthritis; gaps indicate the intra-joint space between the articular surface of the tibia and femur. Scale bar = 80 μm.

**Figure 3:** **BrdU, caspase-3, PARP, and COX-2-immunoreative cells in the tibial and femoral articular cartilage.** Of sham controls **(A, B)**, OA controls **(C, D)**, and the diclofenac sodium **(E, F)** or calcium gluconate 100 mg/kg **(G, H)**, 50 mg/kg **(I, J)** and 25 mg/kg **(K, L)**-treated groups. Changes in the numbers of immunoreactive cells were significantly (*p* < 0.01 or *p* < 0.05) inhibited by treatment with calcium gluconate compared with OA controls. Dark brown staining indicates immunoreactive cells; OA, osteoarthritis. Scale bar = 80 μm.

## Discussion

In the present study, no meaningful changes in body weight and/or weight gain were detected in the groups treated with diclofenac sodium or calcium gluconate compared with the sham and OA controls. Changes in body weight and weight gain in all rats were within the normal range of age-matched rats. OA, also known as a degenerative joint disease, is a type of chronic inflammatory disease. Cartilage damage in OA can lead to edematous changes on the surrounding tissues and a marked increase in the thickness of affected joints [20]. The thickness of operated knees was higher compared with those of sham controls, while these changes were markedly inhibited by treatment with calcium gluconate (50 and 100 mg/kg). The effects of calcium gluconate treatment are likely attributable to its anti-inflammatory properties [15,13].

Increases in maximum extension angles in induced knees were markedly inhibited by 50 and 100 mg/kg calcium gluconate or diclofenac sodium; direct evidence suggests that >50 mg/kg calcium gluconate ameliorates the progression of OA. Joint stiffness was evaluated by measuring the maximum extension joint angle, in which 0° is considered the maximum extension.

The Mankin scoring system is a commonly used histopathological method of detecting articular cartilage injuries [18,19,21]. We found that Mankin scores decreased upon calcium gluconate treatment of both the tibia and femur. Therefore, >50 mg/kg calcium gluconate ameliorated OA-associated cartilage damage. In addition, calcium gluconate treatment (>50 mg/kg) reversed the decreased articular cartilage thickness, as did diclofenac sodium.

Numbers of BrdU-immunoreactive cells were decreased significantly in both the femur and tibia surface articular cartilage of OA controls, indicating marked inhibition of chondrocyte proliferation. However, these changes in the numbers of BrdU-immunoreactive cells were inhibited by treatment with 50 and 100 mg/kg calcium gluconate, unlike diclofenac sodium treatment, after which no marked changes in numbers of BrdU-immunoreactive cells were detected. The degree of facilitation of chondrocyte proliferation induced by calcium gluconate differed from that of the diclofenac sodium treatment; therefore, further studies are needed to better understand the mechanism of action of calcium gluconate. Among the methods of evaluating cell proliferation in histological sections, BrdU immunohistochemistry is the most preferable. In addition, BrdU uptake can be used to evaluate chondrocyte proliferation in OA cartilage [22].

Decreases in the numbers of caspase-3- and PARP-immunoreactive cells among femur and tibia chondrocytes indicate that 50 mg/kg calcium gluconate protects chondrocytes against apoptosis. In addition, the decrease in COX-2-immunoreactivity in the femur and tibia articular cartilage suggests that 50 mg/kg calcium gluconate inhibits COX-2 overexpression. Indeed, it is hypothesized that calcium gluconate exerts anti-inflammatory effects mediated by inhibition of COX-2 expression and related chondrocyte apoptosis. Consequently, calcium gluconate exerted favorable protective effects against OA similar to those of diclofenac sodium. Inhibition of COX-2 and prostaglandin synthesis by traditional NSAIDs and COX-2 inhibitors provides effective relief of OA symptoms [12]. These results indicate that calcium gluconate ameliorates OA via COX-2 inhibition, leading to repression of chondrocyte apoptosis. Increasing evidence suggests the involvement of chondrocyte apoptosis in the pathogenesis of OA [2,8]. Ou et al. reported that celecoxib (a selective COX-2 inhibitor) diminishes OA by repressing chondrocyte apoptosis [13]. In addition, inhibition of COX-2 can reduce the caspase-3 level and chondrocyte death [16].

In the present study, obtaining X-ray images of rats is difficult due to their small size; in general, X-ray analysis and radiological scoring is suitable for larger animals, such as rabbits. Although we identified amelioration by calcium gluconate of OA in rats by histological analysis, further studies using high-resolution X-ray equipment are required to clarify the effect of calcium gluconate on OA.

Taken together, our results indicate that calcium gluconate ameliorates the articular stiffness and cartilage damage associated with OA. Our results suggest that doses of calcium gluconate >50 mg/kg have a protective effect against OA through inhibition of COX-2 overexpression and related chondrocyte apoptosis.

## Conclusions

The results obtained in this study suggest that oral administration of calcium gluconate (>50 mg/kg) for 84 consecutive days ameliorates articular stiffness and cartilage damage compared to OA controls, possibly by inhibiting overexpression of COX-2, a key enzyme in prostaglandin synthesis and related chondrocyte apoptosis. Similar favorable effects on OA-mediated stiffness and cartilage loss were detected in rats that received 50 mg/kg calcium gluconate orally. Moreover, calcium gluconate increased BrdU uptake, based on the numbers of BrdU-immunoreactive cells in both the femur and tibia articular cartilage at 84 days after intra-joint treatment with calcium gluconate.

## Competing interests

The authors declare that they have no competing interests.

## Authors' contributions

S-JK and Y-JL participated in data collection and analysis and wrote the manuscript. J-WK and K-YK produced and supplied calcium gluconate and its material information. S-KK conceived the idea of this study, prepared the protocol, and collected and analyzed the data. All authors read and approved the final manuscript.
